# Application of Intelligent Taste Analysis Based on Random Forest Algorithm in Food Quality Inspection

**DOI:** 10.1155/2022/6901184

**Published:** 2022-07-30

**Authors:** Xinghua Zhang, Yongjie Sun, Yongxin Sun

**Affiliations:** ^1^Changchun Sci-Tech University, Changchun 130600, JiLin, China; ^2^College of Life Science, Changchun Sci-Tech University, Changchun 130600, JiLin, China; ^3^College of Physics and Electronic Information, Baicheng Normal University, Baicheng 137000, Jilin, China

## Abstract

Food safety is a major concern that has an impact on the national economy and people's lives. The food industry has grown in quality and innovation in tandem with the rapid development of the economy and society. The emergence of new food technologies, as well as changes in dietary habits, has increased public concern about food safety. With the emergence of various counterfeit and substandard products, food quality and safety testing have become even more important. Traditional testing methods rely on sensory analysis and physical and chemical analysis. This approach is subjective and poorly adapted to the general public. It requires a high level of technical operation and is difficult to carry out on a large scale. To address this situation, this paper proposes an intelligent approach to food safety quality testing. The core idea is, first, to use sensors to collect data on the various components of the sample to be tested. Second, the random forest (RF) model used in this paper is trained. Third, the trained model is used to classify and identify the test samples. Based on the classification results, a conclusion is drawn as to whether the food product is a variant or a counterfeit. The advantage of this study is that the training model used is a weighted RF algorithm based on mutual information. The correlation between any two decision trees is calculated using mutual information, and for the more correlated decision trees, only the one with the highest evaluation accuracy is retained to form a new RF, and the evaluation accuracy is converted into voting weights, resulting in an RF model with less redundancy and higher evaluation accuracy. The experimental results show that the method used in this paper can successfully identify spoiled or counterfeit products and has good practicality.

## 1. Introduction

Food safety usually means that the items people consume are nontoxic; that is, they do not cause any harm to the body after consumption, and they provide the body with the nutrients it needs [1, 2]. Food safety is not just something that the producer needs to be aware of since there are multiple components involved in the process of food from production to consumption. Food safety is a matter that is jointly guaranteed in many fields. Eating is one of the most important things for human beings. Therefore, food safety and security are of the utmost importance. With the development of technology, many unscrupulous businessmen use high technology to make some poor-quality food products for sale to earn high profits. The packaging of these foods often looks attractive, and the food looks fresh and tasty. In order to achieve the purpose of attracting customers, unscrupulous businessmen will use some ingredients that are toxic and harmful to the human body. And consumers often focus only on the packaging or indication of the food and lack of food safety awareness. Consumers should therefore increase their awareness and knowledge of food safety, develop a healthy and scientific view of consumption, and actively participate in the regulation of food safety to ensure food safety and health. The protection of food safety is the legal responsibility of all food producers and operators, governments at all levels, and relevant regulatory agencies. Regulation should be continuously strengthened to promote a steady improvement in the internal management capacity of producers and operators by enhancing constraints from society. At the same time, the whole community must take an interest in and maintain food safety and support the work of the government. At present, many consumers have little awareness of the importance of safety management in food businesses, knowledge of consumer culture is still lacking, and the basis for social development of food safety is still not strong. When we are in food safety and find illegal problems, we should take positive action and take the initiative to report them to the regulatory authorities, rather than just complaining and grumbling, not to mention creating false information out of thin air, which will only interfere with normal regulatory work and bring about consumer panic, with the ultimate victim being the consumer.

Food quality and safety are very important, and the government is also the introduction of relevant policies to protect the quality of food. The current policy is mainly from the following aspects. The first is to strengthen the quality control of food sources and strict food into the market trading system. Food safety must start at the source, from planting, breeding, production and processing, wholesale and retail, and consumer four links to carry out a full range of supervision. The use of computers and other modern technical means is to establish a series of systems such as commodity labeling and quality tracing. The second is to establish an industry self-regulatory mechanism to ensure food safety. The credit self-regulation of food production and operation enterprises is particularly important to ensure food safety. Therefore, it is necessary to accelerate the construction of a food safety credit system and establish industry credit standards for food distribution enterprises. We should strengthen the legal system construction and integrity education for operators and urge enterprises to improve their awareness of integrity, quality, and legal operation. The third is the establishment of food safety standards and inspection and testing systems. Product and health standards are established comprehensively related to food safety, and a food safety standards system is built. At the same time, the food safety testing system is improved to ensure that the hygienic quality of food listed for sale meets the requirements of health standards. Fourth, a traceability system that can be traced back to the source is established. Food safety is a complex process that must consider all stages of the food chain, from farm to fork.

The government has given a series of safeguards from the production of food to its final consumption in people's mouths. The most important part of the whole safeguarding process is the occasional inspection of food quality. Traditionally, food quality checks have relied on manual inspection by quality inspectors, which is both energy and time consuming and inefficient. As a result, in recent years, smarter methods of food quality inspection have emerged one after another. The core idea is to identify the quality of food by recognizing the taste of the food. Reference [3] proposed an improved K-means algorithm for detecting spoiled food. The core idea of the study is to segment the pictures of food products in order to determine the degree of spoilage. Reference [4] uses deep learning algorithms based on computer vision techniques to detect and analyze the quality of complex food products. Reference [5] devised a relationship between food quality and preservation conditions based on Fourier's law of conduction. Reference [6] proposed a quality inspection technique for frozen foods. The core technique used in this study was Raman spectroscopy. Reference [7] introduced blockchain technology for the storage and preservation of food products, thus guaranteeing food quality and safety. Reference [8] summarizes a variety of deep learning techniques applied to the inspection of food quality such as fruits, vegetables, and meat. Reference [9] uses image processing techniques applied to the detection of egg quality. The study combines hyperspectral imaging, multivariate analysis, and image processing to identify the freshness of eggs as well as the breakage of eggs. Experimental results showed that this aspect was able to achieve a detection rate of over 97%. For quality detection of palletized packaged food, reference [10] used a deep neural network based on a principal component analysis network. Experiments were conducted using support vector machines (SVM) [11] as well as K-nearest neighbours (KNN) [12] for experimental comparison, which showed that the study has advantages not only in terms of detection accuracy but also speed. From the above studies, it can be seen that for food quality inspection, more and more scholars are introducing intelligent algorithms such as machine learning algorithms [13–15] and deep learning [16–18] algorithms. The use of intelligent technologies has indeed improved the efficiency and accuracy of food quality inspection and saved human and material resources. In this paper, RF algorithm is introduced for food quality inspection based on taste analysis. Experiments on vinegar demonstrate the effectiveness of the method in this paper.

## 2. Relevant Knowledge

### 2.1. Taste Analysis Methods

It is well known that the taste signals received by the human brain are produced by taste receptor cells in the mouth (mainly the tongue). These taste receptor cells interact with specific chemicals in food. Different types of taste cells are sensitive to specific flavour substances. This property enables humans as well as animals to recognize different tastes. Early artificial taste systems used generic sensors or methods to recognize the physicochemical properties of food. For example, for salty tastes, they can be measured using conductive agents, and for sour tastes, their pH can be measured directly to characterize the acidity. The most primitive calibrations were obtained using a comparison of the human evaluation of salty and sour flavours and the quantitative values detected by the sensors. AsHumans have vague descriptions of taste, e.g. “a little sour”, “very sour.” The machine, on the other hand, obtains precise measured values. This method therefore only yields results that are not uniform. Later research, towards multisensor multicomponent analytical chemistry methods, which rely on specific chemical sensors, is difficult to implement and difficult to generalize.

On the other hand, there is ongoing research into the underlying perceptual mechanisms of the taste nerve. It has been found that taste cells are not actually sensitive to only one chemical substance but respond to a variety of substances. At the same time, when different taste nerve cells perceive a stimulus at the same time, they transmit their respective signals to the center, which ultimately decides what type of taste stimulus to receive. A diagram of this process is shown in Figure 1. This mechanistic understanding is the cornerstone of modern taste sensing and analysis, resulting in the approach of cross-response sensor arrays. That is, a small number of types of sensors, through a mechanism similar to that of a neural network, are ultimately able to identify a larger number of types of taste stimuli. The number of stimulus types is an order of magnitude greater than the number of sensor types. Importantly, this approach draws on bionic ideas and breaks through the constraints of strongly selective taste sensors.

The traction in this mechanistic understanding has led to a move away from reliance on specific taste sensors for taste sensing. Tests have been carried out using less selective sets of sensors, which are analyzed by chemical analysis methods as well as by pattern recognition methods. This approach allowed pattern recognition to be used naturally in taste recognition scenarios. This was followed by the development of artificial taste sensing. And nowadays, the conceptual definition of taste sensors and electronic tongues and the mathematical processing methods used have gradually become clearer. With the development of materials, computers, and physical-chemical testing techniques, more sensors are available, and the accuracy and range of tests have advanced dramatically. A schematic representation of modern methods of artificial taste analysis is shown in Figure 2.

### 2.2. Application of Taste Analysis Methods

With the rapid development of electronic tongues and taste sensors, the recognition of types of taste is no longer limited to the recognition of simple basic characteristics such as sweet, sour, bitter, spicy, and salty. Application scenarios now include flavour and quality recognition, such as flavour recognition of alcohol and beverages, determination of the quality of liquid and solid foods, and can even be used to distinguish minor differences between different manufacturers' brands of the same type of food. More work has been carried out on the artificial taste analysis of liquid beverages than on the taste analysis of solid foods. A large body of literature deals with, for example, fruit juices, alcoholic beverages, and liquid flavourings. Reference [19] used multiple sensors to capture the composition of red wine in order to correctly differentiate the taste of red wine. Pattern recognition techniques were also used to perform operations such as preprocessing and classification of the collected data from the red wines. The experimental results show that the method used in this literature can successfully identify red wines as well as nonred wines. Reference [20] used a highly cross-selective sensor to capture the composition of red wines and combine it with principal component analysis and clustering algorithms to model and identify changes in the taste of red wines during storage. Reference [21] used an electronic tongue to capture the concentration of bisulphite in wine and trained a prediction model using the PLS method. The results showed that the method was effective in predicting the bisulphite concentration. PLS combined with linear discriminant analysis (LDA) was used in reference [22] to determine the taste of yellow wine (a Chinese rice wine). The data were used to analyze the taste characteristics of yellow wine from various regions.

## 3. Improved RF-Based Food Quality Detection Algorithm

### 3.1. Traditional RF

In the 1980s, Breiman et al. developed the classification tree algorithm, which was much less computationally intensive than repeatedly dichotomizing data for classification or regression. Breiman combined the classification trees into an RF in 2001 by randomly generating many classification trees and then aggregating the classification tree results. RF improves prediction accuracy without requiring significantly more computing power. RF is considered one of the best current algorithms because they are insensitive to multicollinearity. RF can deal with noisy and unbalanced data very well, which is one of the important reasons why the algorithm can be widely used.

RF selects *n* samples from the *N* training samples, which are typically much smaller than *N*, and repeats the process *C* times to generate *C* decision trees. When splitting each node of the decision tree, *d* attributes are chosen at random from all *D* attributes, and the best attribute from the *d* attributes is chosen as the splitting attribute. The CART algorithm is commonly used to select the splitting attributes. The Gini index can determine the splitting attributes in this algorithm. The Gini value of *V* is calculated by (1). Assuming that the proportion of the *i*-th category in the current sample set *V* is *s*_*i*_, where *S*_*i*_ = 1 and *k* denotes the total number of categories.

(1) $$\begin{array}{c} \text{Gini}\left(V\right)=1-\sum_{i=1}^{\left|k\right|}s_{i}^{2}. \end{array}$$

The Gini value is taken to be between 0 and 1. The test attribute *β* is used to dichotomize the random variable *V* into two categories *V*_1_ and *V*_2_, and then, the Gini index for attribute a is calculated as follows:

(2) $$\begin{array}{c} \text{Gini}\left(V,\beta \right)=\frac{\left|V_{1}\right|}{\left|V\right|}\text{Gini}\left(V_{1}\right)+\frac{\left|V_{2}\right|}{\left|V\right|}\text{Gini }\left(V_{2}\right). \end{array}$$

Assuming that the set of candidate attributes is (*B*=*β*_1_, *β*_2_,…, *β*_*d*_), then the attribute that minimizes the Gini index after division is selected as the optimal divided attribute.

(3) $$\begin{array}{c} \beta^{*}=\arg\;\min\left(\text{Gini}\_\text{index}\left(V,\beta \right)\right). \end{array}$$

### 3.2. Improving RF

Traditional RF generates decision trees with high similarity, rendering the trained model obsolete. Furthermore, in the voting process, all decision trees are given the same weight by default, ignoring any differences in performance between different decision trees. To address these issues, this paper proposes IRF that incorporates mutual information and a weighting strategy to optimize the RF. The correlation between any two decision trees is calculated using mutual information, and only the one with the highest evaluation accuracy is retained for the more correlated decision trees, forming a new RF and converting the evaluation accuracy into voting weights to obtain a RF model with less redundancy and higher evaluation accuracy.

Mutual information is used to measure the interdependence between two variables. For two sets of given random variables *X*_1_ and *X*_2_, their mutual information is expressed as

(4) $$\begin{array}{c} MI\left(X_{1},X_{2}\right)=L\left(X_{1}\right)\sum_{x_{1}\in X_{1}}\sum_{x_{2}\in X_{2}}p\left(x_{1},x_{2}\right)\text{log}\frac{p\left(x_{1},x_{2}\right)}{p\left(x_{1}\right)p\left(x_{2}\right)},\\ =L\left(X_{1}\right)+L\left(X_{21}\right)-L\left(X_{1},X_{2}\right), \end{array}$$

where *p*(*x*_1_, *x*_2_) is the joint probability distribution of *X*_1_, *X*_2_, *p*(*x*_1_) and *p*(*x*_2_) are the marginal probability distributions of *X*_1_, *X*_2_, respectively, and *L*(*X*_1_) is the information entropy of *X*_1_, which is calculated as

(5) $$\begin{array}{c} L\left(X_{1}\right)=-\sum_{x_{1}\in X_{1}}p\left(x_{1}\right)\text{log}p\left(x_{1}\right), \end{array}$$

where *p*(*x*_1_) denotes the probability of event *x* occurring; *L*(*X*_2_) is the information entropy of *X*_2_, and *L*(*X*_1_, *X*_2_) is the joint entropy, which is calculated as

(6) $$\begin{array}{c} L\left(X_{1},X_{2}\right)=-\sum_{x_{1}\in X_{1}}\sum_{x_{2}\in X_{2}}p\left(x_{1},x_{2}\right)\text{log}p\left(x_{1},x_{2}\right). \end{array}$$

For a decision tree *l*_*i*_ (*i* = 1, 2, ..., *C*) in a RF, *MI*(*l*_*i*_, *l*_*c*_) (*c* ≠ *i*) represents the mutual information of the decision tree *l*_*i*_ and *l*_*c*_. In this paper, *MI* (*l*_*i*_, *l*_*c*_) (*c* ≠ *i*) is used to calculate the correlation between decision trees *l*_*i*_ and *l*_*c*_. The formula is

(7) $$\begin{array}{c} MI\left(l_{i},l_{c}\right)=MI\left(z_{i},z_{c}\right), \end{array}$$

where *z*_*i*_ (*i* = 1,2, ..., *C*) is the *i*-th decision tree's output state. The greater the value of *MI*(*l*_*i*_, *l*_*c*_), the greater the correlation between the two decision trees, and the greater the degree of information overlap. A group of decision trees with mutual information values greater than a threshold *ε* will be combined by calculating the mutual information of any two decision trees. *MI*(*l*_*i*_, *z*) represents the mutual information between the decision tree *l*_*i*_ and the actual label *z*, that is, the correlation between the decision tree *l*_*i*_'s output evaluation result and the actual evaluation result. The equation is

(8) $$\begin{array}{c} MI\left(l_{i},z\right)=MI\left(z_{i},z\right). \end{array}$$

The larger the value of *MI*(*l*_*i*_, *z*), the higher the evaluation accuracy of the decision tree *l*_*i*_. Finally, the decision trees with less correlation and higher accuracy are formed into an IRF. The steps of IRF implementation are as follows:

1. Step 1: get the training set *X*={(*x*_1_, *y*_1_), (*x*_1_, *y*_1_),…, (*x*_*N*_, *y*_*N*_)}, validation set *X*′={(*x*_1_, *y*_1_), (*x*_1_, *y*_1_),…, (*x*_*L*_, *y*_*L*_)}, *x*_*i*_ is the sample, and *y*_*i*_ is label.
2. Step 2: draw *n* samples from *X* by bootstrap sampling and repeat *T* times to obtain *T* training sets.
3. Step 3: for each internal node of the decision tree, *d* attributes are randomly selected from the sample *D* attributes, and the best splitting attribute among the *d* attributes is chosen as the test attribute of the node.
4. Step 4: generate *T* completely random decision trees to form a RF *R*={*l*_1_, *l*_2_,…, *l*_*t*_}.
5. Step 5: input the validation set X′ into *R* to get the result.
6. Step 6: based on the results, the correlation between each decision tree and the rest of the decision trees is calculated in turn. All the decision trees with *MI*(*l*_*i*_, *l*_*c*_)(*i* ≠ *c*) greater than the threshold *ε* are combined into one decision tree group. If the correlation between *h*, and all other decision trees is less than or equal to the threshold *ε*, then the decision trees are grouped separately.
7. Step 7: repeat step 6 for the out-group decision trees in order until all decision trees are grouped.
8. Step 8: obtain the decision tree with the highest accuracy in each group based on the accuracy *MI*(*l*_*i*_, *z*).
9. Step 9: form a new RF from the obtained decision trees *R*′={*l*_1_′, *l*_2_′,…, *l*_*t*_′}.

When evaluating the input sample data, the traditional RF has the same voting weight for each decision tree, which ignores the influence of the evaluation accuracy of different decision trees on the final result and reduces the evaluation accuracy of the RF as a whole. In order to increase the number of decision trees with high evaluation accuracy and reduce the influence of decision trees with low evaluation accuracy on the final evaluation results, this paper proposes a weighted voting method to convert the evaluation accuracy into the voting weights of decision trees. After the traditional RF is streamlined, the evaluation accuracy matrix *A* of decision trees in the IRF is

(9) $$\begin{array}{c} A=\left[\begin{array}{cccc} a_{11} & a_{11} & \cdots & a_{11}\\ a_{21} & a_{22} & \ddots & a_{2c}\\ \vdots & \vdots & \ddots & \vdots \\ a_{G1} & a_{G2} & \cdots & a_{GC} \end{array}\right], \end{array}$$

where *a*_*gc*_ denotes the evaluation accuracy of the *c-*th decision tree for the *g*-th running state, where *c* = 1,2, ..., *C*, *g*  = 1,2, ..., *G*, *G* is the number of classes of evaluation results, and *C* is the number of improved decision trees which obtained by substituting the validation set *X*′ into IRF and calculating the correctness of the output of each decision tree for each class.

Based on the evaluation accuracy matrix, the weight matrix *Q* is defined as

(10) $$\begin{array}{c} Q=\left[\begin{array}{cccc} q_{11} & q_{11} & \cdots & q_{11}\\ q_{21} & q_{22} & \ddots & q_{2c}\\ \vdots & \vdots & \ddots & \vdots \\ q_{G1} & q_{G2} & \cdots & q_{GC} \end{array}\right], \end{array}$$

where *Q*_*gc*_ is the weight of the *p* th tree for the *g*-th running state, which is calculated as

(11) $$\begin{array}{c} q_{gc}=a_{gc}. \end{array}$$

The specific flow of the IRF is shown in Figure 3.

## 4. Experimental Analysis

### 4.1. Experimental Background

In recent years, there has been an increase in the number of counterfeit and shoddy products. These products often have identical outer packaging, but the quality of the product varies. This paper uses a taste-based food quality detection method. To verify the effectiveness of the method, data from different brands of vinegar are collected and analyzed, and the brands of the respective products are identified. If the results obtained by the RF algorithm for a product captured do not belong to an existing product class, this indicates that there is a problem with the quality of the product. Based on this idea, a Chinese food product vinegar was experimentally analyzed in the experimental part. The evaluation metrics used during the experiments to quantify the effectiveness of the classification models used in this paper are shown in Table 1.

Since the sample size collected during the experiment was not very large, a 5-fold cross-validation method was used to ensure the validity of the experiment, and 60% of the sample overview was selected as the training sample and 40% of the sample as the test sample. The comparison algorithms used were all classical classification algorithms, mainly SVM [23], RF (RF) [24], radial basis function neural network (RBFNN) [25], and Naive Bayes (NB) [26].

### 4.2. Vinegar Quality Inspection Experiment

The taste of different types of table vinegar is different because the raw materials and processes used to make them are different. Edible vinegar is an acidic condiment that is often used when people cook ingredients. Protein, fat, carbohydrates, ash, water, energy, riboflavin, sodium, potassium, calcium, magnesium, iron, manganese, zinc, copper, phosphorus, and selenium are the main components of table vinegar. Leucine, isoleucine, lysine, methionine, cystine, phenylalanine, tyrosine, threonine, tryptophan, arginine, histidine, alanine, valine, glycine, proline, glutamic acid, serine, and aspartic acid are all found in it. In this paper, a total of five types of edible vinegar were selected: white vinegar, rice vinegar, aged vinegar, balsamic vinegar, and sugar vinegar. The quantitative indexes of each edible vinegar are shown in Table 2. *I*1, *I*2, *I*3, *I*4, and *I*5 represent total soluble sugar, total acid, salt, sugar-acid ratio, and pH, respectively. The sugar-acid ratio was determined by averaging total sugar and total acid.

Principal component analysis was conducted on the five component indicators of the above five types of vinegar, and the principal component score plots are shown in Figures 4 and 5. The variance contribution of the first principal component was 56.28 percent, the variance contribution of the second principal component was 25.93 percent, and the cumulative variance contribution of the first and second principal components was 83.54 percent, explaining the majority of the variance. Therefore, the first 2 principal components can only represent 82.21% of the information contained in the original 5 physical and chemical indicators. In addition, the five types of samples could not be well separated on the first principal component score axis, only white vinegar and sugar vinegar could be distinguished from the other types of vinegar, and there was great dispersion between the different brands of rice vinegar, while aged vinegar and balsamic vinegar were seriously confused with each other, which indicated that aged vinegar and balsamic vinegar had some similarity, while white vinegar and sugar vinegar were very different from the other types and showed specificity, and the samples of rice vinegar were more different from each other. It is difficult to group them together because of the relatively large differences between the samples of rice vinegar. This indicates that the first principal component obtained from the physicochemical indicators can be interpreted as the sugar content (sweetness) and that the first principal component is positively correlated with the sugar content. Furthermore, the distribution from left to right is roughly in the ascending order of the sugar-acid ratio, indicating that the first principal component can also be interpreted as the sugar-acid ratio and that the first principal component is positively related to the sugar-acid ratio. On the second principal component score axis, the five types of samples are also differentiated, and intuitively, the five types are distributed on the second principal component score axis from bottom to top in an ascending order of total acidity, which indicates that the second principal component obtained from the physicochemical indicators can be interpreted as acidity (sourness) and that the second principal component is positively correlated with acidity. In general, the results of the principal component analysis obtained from the physicochemical indicators were mainly related to the brix and acidity characteristics of vinegar, which is not unrelated to the fact that vinegar is an acidic condiment. However, these five physicochemical indicators alone are not sufficient to distinguish the different types of vinegar.

Sixty samples were taken from each category of edible vinegar. The total number of samples was 300. Eight indicators were collected for each type of edible vinegar. These 8 indicators were collected by 8 sensors. The size of the samples was 300*∗*8. Since there were 5 types of edible vinegar in total, the number of categories was 5. The results of the experiment are shown in Table 3 and Figure 6.

In terms of recognition accuracy, the IRF method used in this paper improves 0.40, 0.32, 0.27, and 0.10 compared to other SVM, RBFNN, NB, and RF. The improvement ratios fully demonstrate the superiority of this method. In terms of accuracy, the IRF method improves 0.48, 0.47, 0.41, and 0.22 over SVM, RBFNN, NB, and RF, respectively. The high *F*1 scores indicate that the model used in this paper has a good recognition rate for both positive and negative samples. The value range of the four indicators used in this paper is between 0 and 1. The larger the value, the better the performance of the model. The experimental results show that the IRF algorithm has the largest value on the four indicators and is far ahead of other comparison models. The experimental results verify the effectiveness of the IRF algorithm in the detection of edible vinegar quality.

## 5. Conclusion

There have been numerous issues with food quality and safety in recent years. Although the government has introduced relevant policies, it has not been able to eliminate all kinds of counterfeit and shoddy products. On the other hand, many food products are prone to deterioration during storage. If people do not detect these food products in time, they can be harmful to their health. This paper proposes the use of an improved RF algorithm to improve the speed and accuracy of food quality detection. The algorithm uses mutual information to calculate the correlation of any two decision trees, and for the more correlated decision trees, only the decision tree with the highest evaluation accuracy is retained, thus forming a new RF, converting the evaluation accuracy into voting weights, and finally obtaining an RF model with less redundancy and higher evaluation accuracy. The experimental results show that the method used in this paper can successfully identify spoiled or counterfeit products. However, although the algorithm in this paper is more intelligent than traditional food detection methods, there are some problems. One is that the model used does not achieve the desired results for high-dimensional data. Second, it is unknown how well the food testing method proposed in this paper can detect the quality of other food products, as the core ingredients of different food products are different. The determination of the core components has a great impact on the final identification effect. For the above two problems, this paper will be followed by an in-depth study.

## Figures and Tables

**Figure 1:** Nerve center determines taste stimuli.

**Figure 2:** Artificial taste analysis.

**Figure 3:** IRF flow chart.

**Figure 4:** Schematic diagram of principal component analysis of component indicators.

**Figure 5:** Factor loading diagram.

**Figure 6:** Comparison of classification results of different models.

**Table 1:** Introduction to evaluation indicators.

Name	Expressions
Accuracy	Accuracy=(Number of correctly classified samples/total number of samples)
Precision	Precision=(true sample number/true sample number+false positives number)
Recall	Recall=(true sample number/true sample number+false negatives number)
*F*1 score	*F*1=2^*∗*^Precision*∗*Recall/Precision+Recall

**Table 2:** Quantitative indicators for table vinegar.

Index\Type	Vinegar 1	Vinegar 2	Vinegar 3	Vinegar 4	Vinegar 5
*I*1 (%)	3.86 ± 0.57	7.55 ± 0.73	14.51 ± 0.28	14.64 ± 0.63	7.17 ± 0.81
*I*2 (%)	4.82 ± 0.62	6.46 ± 1.03	5.45 ± 0.53	5.35 ± 0.55	4.65 ± 1.02
*I*3 (%)	0.94 ± 0.38	1.28 ± 0.84	1.82 ± 0.44	1.79 ± 0.84	1.42 ± 0.87
*I*4 (%)	0.80 ± 0.92	1.17 ± 091	2.66 ± 0.38	2.74 ± 0.97	1.54 ± 0.53
*I*5	2.53 ± 0.86	2.49 ± 0.40	3.32 ± 0.64	3.54 ± 0.63	3.38 ± 0.62

**Table 3:** Classification results of different models for vinegar.

Model\Index	Accuracy	Precision	Recall	*F*1
SVM	71.49%	67.35%	78.10%	72.33%
RBFNN	75.87%	67.99%	76.25%	71.88%
NB	78.83%	70.89%	71.92%	71.40%
RF	90.53%	81.93%	74.03%	77.78%
IRF	100%	99.83%	96.47%	98.12%

## Data Availability

The labeled data set used to support the findings of this study is available from the corresponding author upon request.
